This article has been retracted.

# Automatic Music Classification Model Based on Instantaneous Frequency and CNNs in High Noise Environment

**DOI:** 10.1155/2022/1317439

**Published:** 2022-09-21

**Authors:** Wen Lai

**Affiliations:** School of Music Jinzhong University, Jinzhong 030600, China

## Abstract

Automatic music classification has significant research implications because it is the foundation for quick and efficient music resource retrieval and has a wide range of possible applications. In this study, DL is used to extract and categorize musical features, and a DL-based model for music feature extraction and classification is created. In this study, the instantaneous frequency and short-time Fourier transform are used to estimate the sine of a mixed music signal. Based on peak-frequency pairs, the DL algorithm is then used to calculate multiple candidate pitch estimates for each frame, and the melody pitch sequence is then obtained in accordance with the pitch profile duration and continuity characteristics. With this approach, the pitch can be calculated without reference to the fundamental frequency component. A music feature classification approach using spectrogram as input data and CNN as classifier is proposed at the same time in light of CNN's benefits in image processing. Studies reveal that this model's categorization and music feature extraction accuracy is as high as 94.18 percent and 95.66 percent, respectively. The outcomes demonstrate the efficiency of this technique for the extraction and classification of musical features. The field of music information retrieval is a good fit for it.

## 1. Introduction

Music is divided into physical music and digital music, in which physical music is stored by physical hardware such as tapes and CDs, while digital music is stored digitally, which can be subdivided into data storage form and streaming media form [1]. Technological progress in music-related fields has prompted digital music to lead the development of music industry. The change of music carrier makes the music information on the Internet show explosive growth, while the massive music data increases the information fatigue of users. How to better classify it has already been put on the agenda, thus leading to music information retrieval. Research in the field of music information retrieval refers to music content analysis, music retrieval, and music recommendation based on modern intelligent information processing technology [2]. The three most frequent categories used to categorize music nowadays are music genre, music emotion, and music appropriate scenario. According to music style, which music elements are used in arrangements, which music qualities are displayed, and different music genres are classified [3]. People can more easily find the music they want by having music classified in a variety of ways because different people have varied requirements for music classification. The preferences of individuals for different musical genres also push service providers to deliver more accurate music classification results. It is essential to employ computer systems to automatically identify music genres because the old method of analyzing music by professionals and classifying it manually cannot handle vast music [4]. The fundamental frequency sequence, spectral square, and amplitude envelope of the music signal are among the physical properties of the digital signal that content-based music retrieval technology investigates. Intermediate characteristics include the melody's rhythm, timbre, and harmony, even more sophisticated features, such as music texture and style [5]. Once these features have been extracted, you can use them as query criteria to look for music that most closely matches the extracted features in a library of preexisting music features.

The classification of music by hand labelling is inefficient and unrealistic in the age of big data. The process of classifying music based on its content often involves manually extracting its features, which are subsequently entered as training data into a model using the machine learning classification approach [6]. Establish a great music index system after appropriately classifying the vast music resources to help people locate the music they want more easily, increase the effectiveness of music retrieval, and then enhance how people search for and enjoy music to bring out the most enjoyment from it. In recent years, DL (deep learning) [7] was seen to take the lead in AI development, and CNN (convective neural network) [8, 9] is exceptional in recognising images. With plenty of space for accuracy improvement and good processing efficiency for high-dimensional data, it can effectively identify the features of complex images. Additionally, its architecture and individual components are still evolving quickly. The method of applying DL model in music classification has started to emerge as a result of the widespread application of DL model in other fields. However, there are still several issues with the accuracy, model complexity, model training, and other aspects of the current approaches that require improvement.

In this study, DL is used to extract and categorize musical features, and a DL-based model for music feature extraction and classification is created. The following are its innovations: (1) In this study, music is first preprocessed using the discrete Fourier transform, and then feature vectors are extracted in accordance with the statistical patterns of various musical genres. Finally, a music feature classification approach based on NN (neural network) [10] is constructed. CNN is utilised to train feature vectors. CNN can also automatically pick up abstract features and blend local musical features to create a global statement. (2) This paper designs a complete architecture from input to output and builds a CNN classification model based on spectrogram. In the dynamic planning stage, the rough estimation result of melody contour is smoothed to obtain the dynamic range of melody pitch at frame level, and then the objective function describing the melody pitch is iteratively solved by the dynamic programming algorithm to obtain the final melody pitch sequence. Experimental results show that this method has high accuracy of feature extraction.

## 2. Related Work

In the area of music information retrieval, feature extraction and categorization are a crucial subject, and numerous academics have investigated it and produced significant advancements. The majority of solutions, however, fall short of actual performance requirements, and other issues still need to be investigated and resolved.

Das and Satpathy used CNN to extract multiple features from music signals and classify them [11]. Experiments on the GTZAN dataset show that this method can effectively improve music style recognition using a single feature. Nam J et al. proposed a main melody extraction method combining the improved Euclidean algorithm and dynamic programming [12], aiming at the problem that the pitch estimation value sometimes jumps violently within the same note duration. This method uses the improved Euclidean algorithm to estimate multiple candidate pitches in each frame and uses the dynamic programming algorithm to iteratively solve the objective function describing the pitch of the main melody, so as to obtain a smooth pitch profile of the melody and greatly reduce the short-term sharpness of the melody profile, jump. The experimental results show that the method can effectively estimate the main melody pitch when the fundamental frequency is lost and avoid the short-term violent jump of the melody pitch sequence. Chen and Wang improved the two key steps of feature extraction and classification method based on auditory characteristics and proposed a music classification method based on auditory characteristics CNN for music classification tasks [13]. Aiming at some deficiencies of traditional classification methods, Hadjidimitriou and Hadjileontiadis proposed a pop music classification method based on feature extraction and NN [14]. In terms of feature extraction, this method uses frame energy and frame energy ratio as feature vectors in two music time-domains; finally, BP network is used as a classifier to classify music. Reljin and Pokrajac proposed a retrieval method that considers both pitch and rhythm in their system [15]. Zubair et al. proposed a heuristic-based melody channel selection algorithm, which filters some channels that may contain melody in obvious steps and selects the appropriate channels to combine on this basis and the notes that constitute the melody come from these channels [16]. Saari et al. drew on the two important CNN architectures in the field of computer vision, DenseNet and Inception structure, and proposed a new CNN structure Dense Inception module; and based on this, they proposed a new CNN architecture of dense inception network for music genre classification [17]. Based on the idea of DL and the structural characteristics of CNN, Vyshnav et al. designed a music genre classification model with spectrogram as input, which provided a new idea of audio classification and recognition [18]. Rosner and Kostek compared CNN-based methods with traditional machine learning classification methods [19]. The experimental results show that the CNN-based method is superior to the traditional machine learning classification method in classification accuracy. George and Shamir pointed out that based on the auditory characteristics, CNN divides the time-frequency features of music into different regions according to the frequency and only shares the convolution kernel in the specified region, so that the convolution kernels in different frequency regions can learn the regions feature [20].

This study thoroughly examines the pertinent literature, outlines its benefits and drawbacks, and then proposes a music feature extraction and classification model based on DL. In this research, a CNN classification model based on spectrogram is created, and a whole architecture is designed from input to output. The use of CNN's very effective and potent feature learning and classification capability reduces the time and expense of manual processing. To determine the dynamic range of the melody pitch at the frame level, the rough estimation result of the melody contour is smoothed during the dynamic planning stage. Next, the dynamic programming algorithm solves the objective function describing the melody pitch iteratively to produce the final melody pitch sequence. According to experimental findings, this strategy can significantly increase the precision of music feature extraction and classification.

## 3. Methodology

### 3.1. Music Signal and Spectrum Analysis and DL Basis

The varieties and scope of music that are available to people are constantly expanding due to the rapid development of the digital music industry, the Internet, and mobile devices. Analysis of musical content, classification of musical genres, humming recognition, and music recommendation are all included in the retrieval of musical information. In recent years, it has seen widespread use in a variety of industries, including network music, mobile devices, consumer electronics, games, and entertainment. The identification and classification of music genres are currently the main research areas in music information retrieval. Different genres of music can be categorized according to their hierarchical structures, accompanying instruments, and other elements [21]. Different styles and accompanying instruments also differ from one another. Music genre identification is to label messy music according to the characteristics of each genre. The classification of musical feelings is based on the rhythm, lyrics, and emotions of music. Classification of applicable music scenes is to classify applicable scenes according to the rhythm and instruments of music. In addition, automatic music generation is a research direction developed along with DL in recent years. The so-called automatic music generation is to use DL technology to learn various features of music from a large amount of music data and then automatically generate music by using trained models. If the computer can realize the analysis and retrieval based on audio content, it can reduce a lot of manpower tagging costs, which is of great significance to music creation, dissemination, accurate personalized recommendation, and so on. After the machine learning method is introduced, the possible acoustic features are initially determined by artificial judgment, and these features in music are extracted to train the classifier, thus realizing music classification. However, this kind of method is unstable and needs to design feature sets manually, so it depends on personal experience and professional knowledge to some extent, so the accuracy is difficult to improve.

The traditional manual retrieval method cannot satisfy people's retrieval and classification of massive music information. Music classification is essentially a problem of pattern recognition, which mainly includes two aspects: feature extraction and classification. With the development of big data, people can use more data to train deeper and more complex NN, so as to obtain a higher level of feature learning ability and model generalization ability [22]. After enhancing its architecture and parameters, the deep NN developed from shallow networks like perceptrons, and it is now the cornerstone of deep learning (DL). An artificial NN-based algorithm called DL is employed to study data representation, finding hidden features in data by combining DL low-level features to create abstract high-level features. It is a crucial division of CNN NN. It specialises in processing information with a similar grid structure, such as images, which have a traditional two-dimensional grid. CNN processes input images on multiple levels while extracting advanced feature representations. CNN has robust feature learning and feature extraction capabilities. Convolution operation, pooling operation, and activation function are the three fundamental components of CNN. The DL model is shown in Figure 1.

Sound data storage also has its fixed storage format. There are many types of sound files currently in use. At present, there are some common files: WAV files, VOC files, MIDI files, CD files, MP3 files, WMA files, etc. The frequency spectrum of a note generally includes a fundamental wave and several harmonic components, and the frequency of the fundamental wave is called the “fundamental frequency.” The energy of notes is determined by the amplitude of fundamental and harmonic components, which is one of the main bases of the existing main melody extraction methods. Sound is a kind of mechanical wave, so it is a kind of continuous signal in the process of propagation, that is, the mathematical form in time-domain is a continuous function. But for the human ear, a natural Fourier converter, the sound will be automatically converted into a digital signal after being received. Loudness, pitch, and timbre are the three basic characteristics of sound signals. Pitch, loudness, duration, timbre, and spatial position constitute the basic dimensions of sound. Pitch is the sense of hearing to the level of sound. Pitch estimation, also called pitch estimation or pitch detection, is one of the key technologies in speech, audio, and music information processing. Music is essentially a combination of vibration waves with different frequencies, amplitudes, and phases at different time points. When it is reflected in people's auditory feeling, it will get loudness, tone, melody, timbre, and interval. Further analysis is reflected in the characteristics of melody, rhythm, chord, harmony, emotion, style, and so on. The diversity of these elements and characteristics is the expression of musical differences. Time-domain-based analysis method directly uses the time-domain waveform of sound signal to analyze the characteristics of short-inch average energy or short-inch average amplitude, zero-crossing rate, short-term correlation function, and short-term average amplitude difference function of language signal. The method based on frequency domain is to analyze the frequency domain characteristics of sound, including frequency spectrum, power spectrum, and cepstrum. Music melody extraction is used to generate the frequency sequence values corresponding to the melody pitch of music segments. Besides the main melody component, there are abundant accompaniment components in music, among which percussion instruments have broadband unstructured spectrum. When its energy is not particularly prominent, it has little influence on the extraction of the main melody, while the accompaniment and singing of orchestral instruments have typical harmonic structures. It is challenging to accurately estimate the melody pitch sequence from these tones by computer.

### 3.2. DL-Based Music Feature Extraction and Classification Model Construction

Generally, music is divided into gentle part and climax part, and the climax part is basically what determines the music style. The extraction of features such as the time, frequency, and intensity of climax can be regarded as a classification process. We classify each frame and extract the high tide part and the relatively intense frame as feature vectors. Generally, musical tone signals have fundamental frequency and harmonic components. However, occasionally, the fundamental frequency component cannot be detected because of strong bass accompaniment or some special singing skills, so the method of directly searching the fundamental frequency is not the best solution. However, in addition to the fundamental frequency, there are abundant harmonic components located at integer multiples of the fundamental frequency. Time-frequency analysis is the extension of spectrum analysis, which is more intuitive than spectrum analysis. When analyzing audio signals based on short-time Fourier transform, a window function should be added at each sampling time point. This process is called framing and windowing. After that, the discrete Fourier transform is carried out, and finally, the results generated by the whole signal are stacked, so that the time-frequency distribution diagram of the signal can be obtained, which is a kind of frequency spectrum diagram. The whole process transforms the one-dimensional sound signal into a two-dimensional signal which can reflect the frequency distribution and change with time. On mel-frequency, the distribution of auditory characteristics of human ear is nearly linear. In order to simulate the nonlinear characteristics of human auditory perception and improve the performance and accuracy of music signal feature extraction, mel-frequency cepstral coefficients first divided mel-frequencies based on auditory perception at equal intervals and then mapped them to common frequencies to obtain the center frequency of each filter. The CNN structure of music feature extraction and classification is shown in Figure 2.

Two issues must be resolved in order to use the Fourier transform in digital signal processing: (1) *f*(*t*) for the Fourier transform in mathematics is a continuous signal, while the computer processes digital signals. (2) The concept of infinity is used in mathematics, and the computer can only perform limited times calculation. Usually, people call this the restricted Fourier transform and discrete Fourier transform. The complex matrix of time-frequency phase is obtained by a short-time Fourier transform of audio, and the amplitude spectrum is converted into power spectrum, and the short-time Fourier transform spectrogram is obtained. The audio frequency is transformed by CQT and converted into power spectrum to obtain a constant Q spectrum. The audio frequency is processed by extracting the features of mel-frequency spectrum and visualization to obtain the mel-frequency spectrum. Instantaneous frequency method is often used to obtain accurate sinusoidal frequency estimation, so this method intends to adopt instantaneous frequency method to improve the accuracy of sinusoidal estimation. Parameter sharing means that the convolution kernel is shared in convolution operation, that is, the outputs at different positions are all the same convolution kernel acting on different input areas. Compared with traditional NN parameter sharing, parameter sharing can significantly reduce the number of parameters. At the same time, parameter sharing ensures that CNN only needs to learn one parameter set, instead of learning a separate parameter set for each output unit. The input of this CNN is 288 × 288, but the smaller common resolution is not adopted. The reason is that this network is only used as a 10-classification model, which is very few compared with the 1000 classification of VGG-16. Increasing the resolution of the input picture can increase the amount of information input into the network and improve the classification accuracy when the network depth is sufficient. As a small classification model, it will not increase too much computational burden. Max pooling is used in pooling layer, and both convolution layer and pooling layer appear alternately in CNN.

In digital audio and music signal processing, the centroid of the spectrum is frequently used as a measure of music timbre since it can more accurately reflect the brightness of sound. It has the following mathematical definition:

(1) $$\begin{array}{c} C_{t}=\frac{\sum_{n=1}^{N}M_{t}\left[n\right]\times n}{\sum_{n=1}^{N}M_{t}}, \end{array}$$

where *M*_*t*_[*n*] represents the amplitude of the Fourier transform of the *t*th frame at the frequency group *n*. The timbre of an audio stream or whether it is articulated is typically determined using spectral flux. It has the following mathematical definition:

(2) $$\begin{array}{c} F_{t}=\overset{N}{\underset{n=1}{\sum }}\left(N_{t}\left[n\right]-N_{t-1}\left[n\right]\right). \end{array}$$

The mel-frequency scale corresponds to the auditory properties of the human ear. mel-frequency and frequency *f* have the following relationship:

(3) $$\begin{array}{c} f_{mel}=25951g\left(1+f/700\right), \end{array}$$

where *f*_*mel*_ is the converted mel-frequency, *f* is the frequency, and the unit is Hertz. Assuming that a continuous sound signal *f*(*t*) is uniformly sampled with an interval Δ*t*, the discretization is:

(4) $$\begin{array}{c} \left\{f\left(\left(t_{0}\right),f\left(t_{0}+\Delta t\right),\cdots ,f\left[t_{0}+\left(N-1\right)\Delta t\right]\right)\right\}. \end{array}$$

Represent the sequence as:

(5) $$\begin{array}{c} f\left[n\right]=f\left(t_{0}+n\Delta t\right), \end{array}$$

where *n* is the discrete value 0, 1, 2, 3, ⋯, *N* − 1. So the sampled discrete Fourier transform expression is:

(6) $$\begin{array}{c} F\left(k\right)=\frac{1}{N}\overset{N-1}{\underset{n=0}{\sum }}f\left(n\right)e^{-j2\pi kn/N}, \end{array}$$

(7) $$\begin{array}{c} f\left(n\right)=\frac{1}{N}\overset{N-1}{\underset{n=0}{\sum }}f\left(k\right)e^{j2\pi kn/N}. \end{array}$$

Expression (6) shows that when the computer processes the finite sequence, the signal is processed as a periodic signal, and the period is the same as that of *f*(*n*). Period *T* = *N*. So for an audio file with *N* samples, the size of the periodic Fourier transform is still *N*.

How closely the model's predicted value matches the actual value is determined using the loss function. The resilience of the model is improved via a reduced loss function. If linear regression is used for sample (*x*_*i*_, *y*_*i*_)*i* = 1, 2, 3, ⋯, *m*, its loss function is:

(8) $$\begin{array}{c} J\left(\theta_{0},\theta_{1}\right)=\overset{m}{\underset{i=1}{\sum }}{\left(h\theta \left(x_{i}\right)-y_{i}\right)}^{2}, \end{array}$$

where *x*_*i*_ represents the *i*th sample feature, *y*_*i*_ represents the output corresponding to the *i*th sample, and *hθ*(*x*_*i*_) is the hypothesis function. The network contains *m* neurons corresponding to *m* types of music styles, and the output probability is:

(9) $$\begin{array}{c} p={\left[P_{1},P_{2},P_{3},\cdots ,P_{m}\right]}^{T}. \end{array}$$

Use the Softmax regression formula as follows:

(10) $$\begin{array}{c} p_{j}=\frac{\exp\left(X_{8}^{j}\right)}{\sum_{i=1}^{m}\exp\left(X_{8}^{i}\right)}, \end{array}$$

(11) $$\begin{array}{c} j=1,2,3,\cdots ,m, \end{array}$$

where *X*_8_ is the input of the Softmax function, *j* is the current class being computed, and *p*_*j*_ represents the true output of the *j*th class.

By framing audio, windowing, doing a frame-by-frame Fourier transform, and converting with a mel-scale filter bank, the mel-power spectrum can be generated. The mel-power spectrum calculations serve as the foundation for the computation of mel-frequency cepstral coefficients. First, the mel-power spectrum is transformed into decibels, and then the discrete cosine transform is used to get the mel-frequency cepstral coefficients. The generalization efficiency and resilience of CNN are enhanced by scale invariance, which guarantees that the final output results of this feature are consistent after pooling even if a slight scale change happens in the input. Data augmentation will be used because there is not much training data. The photos from the training set will be randomly stretched, translated, and flipped at the start of each round before being fed into the network. The output will then be compared to the original input without data improvement. Because the penalty factor of pitch difference between adjacent frames is introduced in dynamic planning, it can reduce the situation that the estimated value switches between different notes in the same note duration. Moreover, in dynamic planning, the saliency function is defined based on the pitch of each frame, which can avoid the disadvantage that it is difficult to accurately describe the salient features of pitch profile.

## 4. Result Analysis and Discussion

This section will conduct experiments using the GTZAN dataset in order to assess how well the CNN model performs. It will also analyze performance differences brought on by various network structures and compare the accuracy with other machine learning algorithms that have historically been used for feature extraction and classification from music. 10 musical genres are included in this data collection. They are pop music, reggae, jazz, metal, hip-hop, country, classical, blues, and country music. There are 100 audio files, each lasting 30 seconds, for each musical genre. The dataset for this study is split into three sections: the training set, the verification set, and the test set.  Table 1 displays the experiment's hardware and software configuration.

In this paper, 50% cross-validation is carried out, and Adam is used as the gradient descent optimization algorithm for model training. Because audio contains too much data information, directly as training data, it will lead to a serious shortage of memory. Therefore, it is necessary to extract features that can represent music characteristics from audio files. Among the commonly used music features, this paper selects three features: mel-cepstrum coefficient, spectrum centroid, and spectrum contrast. Firstly, the experimental test data is used to enhance the impact on the classification accuracy of the model. The experimental results are shown in Figure 3.

The experimental findings demonstrate that data improvement can significantly increase the model's classification accuracy. Data enhancement is employed by default in the following experiments in this chapter since it can directly improve the amount of features that the model can learn, especially for small-scale datasets, and there is no evident downside other than lengthening the training time. The network training and optimization process can be completed by using CNN to construct the network model, loss function to measure the classification outcomes of network output, and parameters of the network model to be updated by minimizing the loss function. The experiment makes use of the test set, and Figure 4 displays the test set's mistake.  Figure 5 displays the test set's accuracy.

The training process of the network is transformed into the optimization problem of minimizing the loss function by adjusting the parameters. A good optimization algorithm has the following advantages: speeding up the training rate of the network, shortening the convergence time of the network, and improving the accuracy of the network. Because the features extracted from the data preprocessing part include MFCC, spectral contrast, and spectral centroid, the minimum dimension of these features is 13, and the maximum dimension is 33. Therefore, the number of neurons in the input layer will be different with different feature combinations, and its range is 13-33. The accuracy of training set and test set changes with epoch as shown in Figure 6.

Since NN has a large number of parameters, a large amount of data must be collected in order for the trained model to perform well in generalization. By using a nonrepetitive random sample strategy, the dataset in this experiment is split into independent training set and verification set. The training set's data size is 80,000, whereas the verification set's data size is 10,000. The network model training is finished when the training set data is used as the network model training's input. The accuracy results of feature classification of the model are shown in Figure 7.

The validation set data is used as the input of network model performance test, and then the evaluation of network model performance is completed. Select accuracy as the performance index. The experimental results are shown in Table 2.

Detailed analysis of the data in the table shows that the performance of this model is better than that of the comparison model. Scale invariance ensures that the final output results of this feature are consistent after pooling even if a small amount of scale transformation occurs in the input, which improves the generalization performance and robustness of CNN.

## 5. Conclusions

Traditional music information retrieval mostly uses text and ignores the auditory aspect of music; nevertheless, writing cannot adequately describe the pitch, timbre, and rhythm of music. Automatic music classification has significant research implications because it is the foundation for quick and efficient music resource retrieval and has a wide range of possible applications. In this study, DL is used to extract and categorize musical features, and a DL-based model for music feature extraction and classification is created. First, the convolution kernel is employed from top to bottom, and the input layer and convolution kernel are developed, which makes it simpler for CNN to extract high-level feature data from the spectrum. When data is entered into the network, data enhancement is used, and trials have shown that it is effective. The music is simultaneously preprocessed using the discrete Fourier transform, and the feature vectors are then retrieved in accordance with the statistical guidelines for various musical genres. Finally, a music feature classification approach based on NN is constructed, and feature vectors are trained using CNN. The accuracy of this model's music feature extraction and classification, according to experimental data, is as high as 95.66 percent and 94.18 percent, respectively. The accuracy of music feature extraction and categorization is considerably improved by this technique. There are still several issues with this study, notwithstanding the research findings. Explore the corresponding basic melody extraction techniques, uncover the underlying characteristics of music signals, and learn how timbre and melody relate to other musical elements.

## Figures and Tables

**Figure 1:** DL model.

**Figure 2:** CNN structure of music feature extraction and classification.

**Figure 3:** Data enhancement experiment results.

**Figure 4:** Error result of test set.

**Figure 5:** Accuracy result of test set.

**Figure 6:** Graph of accuracy of training set and test set changing with epoch.

**Figure 7:** Accuracy results of feature classification.

**Table 1:** Setting of experimental parameters.

Project	Set up
CPU	Intel i7-6700
Random access memory	32 GB
Hard disc	SSD 1 TB
Graphics coprocessors	GeForce GTX 1080 Ti
Operating system	Window 10
DL framework	TensorFlow + Keras
Digital signal processing software	MATLAB
Data processing, other software	Python, NumPy

**Table 2:** Evaluation results of network model performance.

Experiment number	Characteristic	Network model	Accuracy (%)	Standard deviation (%)	Running time (s)
1	MFCC	BP model	76.87	8.94	0.094
2	MFCC	LSTM model	81.24	8.64	0.176
3	MFCC	CNN model	94.31	7.51	0.217
4	CFCC	BP model	78.02	6.98	0.087
5	CFCC	LSTM model	82.57	6.05	0.146
6	CFCC	CNN model	95.66	5.37	0.251

## Data Availability

The data used to support the findings of this study are available from the corresponding author upon request.

## References

[1] Corrêa D. C., Rodrigues F. A. (2016). A survey on symbolic data-based music genre classification. *Expert Systems with Applications*.

[2] Wang D., Deng S., Xu G. (2018). Sequence-based context-aware music recommendation. *Information Retrieval*.

[3] Cai X., Zhang H. (2022). Music genre classification based on auditory image, spectral and acoustic features. *Multimedia Systems*.

[4] Dorochowicz A., Majdańczuk A., Hoffmann P., Kostek B. (2017). Comparison of classification of musical genre obtained by subjective tests and decision algorithms. *The Journal of the Acoustical Society of America*.

[5] Wang X. (2018). Research on the improved method of fundamental frequency extraction for music automatic recognition of piano music. *Journal of Intelligent and Fuzzy Systems*.

[6] Cai W., Gao M., Jiang Y. (2022). Hierarchical Domain Adaptation Projective Dictionary Pair Learning Model for EEG Classification in IoMT Systems. *IEEE Transactions on Computational Social Systems*.

[7] Huang Y., Cheng L., Xue L. (2022). Deep adversarial imitation reinforcement learning for QoS-aware cloud job scheduling. *IEEE Systems Journal*.

[8] Zhao M., Chang C. H., Xie W., Xie Z., Hu J. (2020). Cloud shape classification system based on multi-channel CNN and improved FDM. *IEEE Access*.

[9] Ding Y., Zhang Z., Zhao X. (2022). Self-supervised locality preserving low-pass graph convolutional embedding for large-scale hyperspectral image clustering. *IEEE Transactions on Geoscience and Remote Sensing*.

[10] Ning X., Tian W., Yu Z., Li W., Bai X., Wang Y. (2022). HCFNN: high-order coverage function neural network for image classification. *Pattern Recognition*.

[11] Das S., Satpathy S. (2021). Multimodal music mood classification framework for Kokborok music. *Solid State Technology*.

[12] Nam J., Choi K., Lee J., Chou S. Y., Yang Y. H. (2019). Deep learning for audio-based music classification and tagging: teaching computers to distinguish rock from Bach. *IEEE Signal Processing Magazine*.

[13] Chen J., Wang C. (2013). Automatic music stretching resistance classification using audio features and genres. *IEEE Signal Processing Letters*.

[14] Hadjidimitriou S. K., Hadjileontiadis L. J. (2013). EEG-based classification of music appraisal responses using time-frequency analysis and familiarity ratings. *IEEE Transactions on Affective Computing*.

[15] Reljin N., Pokrajac D. (2017). Music performers classification by using multifractal features: a case study. *Archives of Acoustics*.

[16] Zubair S., Fei Y., Wang W. (2013). Dictionary learning based sparse coefficients for audio classification with max and average pooling. *Digital Signal Processing*.

[17] Saari P., Fazekas G., Eerola T., Barthet M., Lartillot O., Sandler M. (2016). Genre-adaptive semantic computing and audio-based modelling for music mood annotation. *IEEE Transactions on Affective Computing*.

[18] Vyshnav M. T., Sachin Kumar S., Mohan N., Soman K. P. (2020). Random Fourier feature based music-speech classification. *Journal of Intelligent and Fuzzy Systems*.

[19] Rosner A., Kostek B. (2018). Automatic music genre classification based on musical instrument track separation. *Journal of Intelligent Information Systems*.

[20] George J., Shamir L. (2014). Computer analysis of similarities between albums in popular music. *Pattern Recognition Letters*.

[21] Lim S. C., Lee J. S., Jang S. J., Lee S. P., Kim M. (2012). Music-genre classification system based on spectro-temporal features and feature selection. *IEEE Transactions on Consumer Electronics*.

[22] Ren J. M., Wu M. J., Jang J. S. R. (2015). Automatic music mood classification based on timbre and modulation features. *IEEE Transactions on Affective Computing*.

